The article "Efficient Synchronous Real-Time CADe for Multicategory Lesions in Gastroscopy by Using Multiclass Detection Model" was published in 2022. Journal: Biomed Res Int.

# Efficient Synchronous Real-Time CADe for Multicategory Lesions in Gastroscopy by Using Multiclass Detection Model

**DOI:** 10.1155/2022/8504149

**Published:** 2022-08-31

**Authors:** Yiji Ku, Hui Ding, Guangzhi Wang

**Affiliations:** Department of Biomedical Engineering, School of Medicine, Tsinghua University, Beijing 100084, China

## Abstract

Often more than one category of lesions in patients' gastrointestinal tracts need to be found in the endoscopic examination. Therefore, there is a need to establish an efficient synchronous real-time computer-aided detection (CADe) system for multicategory lesion detection. This paper proposes to build a system with a multiclass detection model based on the YOLOv5 to detect multicategory lesions synchronously in real-time. Two joint detection CADe systems using multiple single-class detection models with the same structure in parallel or series are established for comparison. A retrospective dataset containing 31117 images from 3747 patients is used in this study. To train the model, various online data augmentation methods and multiple loss functions are used. The proposed CADe system can synchronously detect cancers, gastrointestinal stromal tumours, polyps, and ulcers from different quality input images with 98% precision, 89% recall, and 90.2% mAP. The detection speed is 47 frames per second with a 0.04 s latency on a PC workstation. Compared to the two joint detection CADe systems, the proposed system is more accurate with faster speed and lower latency. Two extra experiments indicated that the lesion detection model based on YOLOv5x could provide better performance than other common YOLO structures and that different accuracy metrics and lesion categories have different requirements for the number of training images. The proposed synchronous real-time CADe system with the multiclass detection model can detect multicategory lesions with high accuracy and speed and low latency on limited hardware. It expands the clinical application of CADe in endoscopy and uses expensive labelled medical images more efficiently than multiple single-category lesion models for joint detection.

## 1. Introduction

Diseases of the gastrointestinal tract are common in humans [1]. Early examination and treatment can significantly improve their effects [2]. The endoscope is the main instrument used to diagnose and treat gastrointestinal lesions in a clinic [3]. Owing to the large number of images generated during the endoscopy, finding all the lesions accurately and timely is difficult. Using computer-aided detection (CADe) system to assist doctors in endoscopy can reduce the rate of misdiagnosis and increase the rate of detection to improve efficiency [4].

The article "Efficient Synchronous Real-Time CADe for Multicategory Lesions in Gastroscopy by Using Multiclass Detection Model" was published in 2022. Journal: Biomed Res Int.

Classical CADe systems mainly use the active-window method with artificially designed features [5, 6]. However, it is unreliable and time-consuming to extract complex pathological features. Deep learning has better feature extraction and classification capabilities [7–9]. It significantly improves the performance of CADe systems [10]. Nowadays, CADe in endoscopy can accurately detect single category lesions in real-time using deep learning models [11–14].

However, there may be more than one category of lesions in a patient's gastrointestinal tract, which should be detected during an endoscopy [15]. This requires the CADe system to detect multiple lesion categories synchronously in real-time. Using multiple single-category lesion detection models parallelly or serially to compose such a system will further raise the hardware requirements with the increase of lesion category without a limit for real-time detection. This will in turn increase the system's building cost. A multicategory lesion detection model may have better detection speed and latency with limited hardware resources. However, whether it can obtain similar accuracy or not remains unanswered. YOLO is a series of one-stage detection models with a good balance between speed and accuracy [16]. These models have shown good performance in single-category lesion detection under endoscopy [13, 14, 17–19]. However, a detailed study on the synchronous real-time detection of multicategory lesions is required.

This paper proposes a scheme to use a multicategory lesion detection model based on YOLOv5 [20] to establish a multicategory lesion CADe system. It can realize synchronous low-delay real-time detection in limited hardware resources. The study also tested two CADe systems for multicategory lesion joint detection using multiple single-category lesion detection models with the same structure. The models used in all three systems are trained on a large and complicated local dataset. Compared with the two joint detection systems, the proposed system obtains better speed and latency on a PC workstation and achieves higher accuracy, which proves that using a multicategory lesion detection model is more effective for detecting multicategory lesions in expensive endoscopic images. To the best of our knowledge, this is the first study on synchronous real-time multicategory detection for gastroscopy. It can help researchers establish more efficient CADe systems for endoscopy.

## 2. Materials and Methods

### 2.1. Dataset

A large and complicated dataset was collected from the hospital for retrospective study in this work. It contains 31117 images from 3747 patients without private information. Experienced doctors manually annotate 27241 lesions in images into four categories: cancer, ulcer, polyp, and gastrointestinal stromal tumour (GIST). The number of images and lesions are shown in Table 1. All images are unmodified and taken by multiple operators using Olympus 260 series endoscopes. The sizes, aspect ratios, and quality of these images are not selected. Some examples of low-quality images in the dataset are shown in Figure 1. The annotated bounding box (bbox) area ratios also have a significant difference. Due to the statistic of the ratio of the target bbox over the entire image area in the dataset, the ratio less than 0.04 is defined as the little target, and the ratio greater than 0.25 is defined as the large target, and the rest are medium targets. The distribution of targets is shown in Figure 2. Such a dataset makes the model more difficult to train but more robust in reality.

The article "Efficient Synchronous Real-Time CADe for Multicategory Lesions in Gastroscopy by Using Multiclass Detection Model" was published in 2022. Journal: Biomed Res Int.

The images in the dataset are numbered and assigned to a training set, validation set, and test set according to the archiving order. The training set contains 3600 images of each category lesion and 3600 negative samples, a total of 18000 images. The validation set contains 1200 images of each image type, totalling 6000 images. All the other 7117 images are included in the test set. The distribution of the category of lesions in these sets is shown in Figure 3, which can be considered balanced. Negative samples included in the dataset ensure that the model would not be overconfident, which is confirmed by other studies [21].

### 2.2. Synchronous Multicategory Lesion Detection System

The proposed multicategory lesion detection system (MDS) is shown in Figure 4. It can synchronously detect cancers, polyps, GISTs, and ulcers in gastroscopy. This system can also obtain low latency and high FPS using limited hardware resources.

Single images are streamed into a YOLOv5-based multiclass detection model (MDM, see Figure 5) to detect multicategory lesions after being preprocessed by scaling and padding to 640 × 640. The HardSwish function [22], expressed in Equation (1), is used as an activation function in the model. The model outputs prediction vectors containing the corner coordinates of detected bboxes of lesions, the categories of lesions, and the confidence scores. IoU-based non-maximum suppression is used to postprocess the prediction vectors. The system converts the vectors into bboxes, selects the one with the highest confidence from multiple overlapping bboxes as the final result, and draws it in the image.

(1) $$\begin{array}{c} \text{HardSwish}\left(x\right)=x\frac{\min\left(6,\max\left(0,x+3\right)\right)}{6}. \end{array}$$

The article "Efficient Synchronous Real-Time CADe for Multicategory Lesions in Gastroscopy by Using Multiclass Detection Model" was published in 2022. Journal: Biomed Res Int.

### 2.3. Multicategory Lesion Joint Detection Systems

MDS is compared with multiple single-category lesion detection models to detect multicategory lesions jointly. A single-class detection model (SDM) is trained for each lesion category. Four SDMs are run parallelly or serially to replace the MDM in MDS to obtain two modified systems. According to the running order of SDMs, the two systems are named multicategory lesion parallel detection system (MPDS) and multicategory lesion serial detection system (MSDS). The system runs SDMs parallelly for MPDS and serially for MSDS to generate prediction vectors. Running *N* SDMs in parallel needs *N* times the computing resources of one model to obtain similar speed and latency. Running *N* SDMs in series needs the same computing resources as one model but nearly *N* times the running time and latency. The preprocessing and postprocessing in the two systems are identical to MDS.

### 2.4. Training Strategy for the Lesion Detection Model

All the systems are implemented on Python 3.8 and PyTorch 1.8, and the models are trained on a workstation equipped with NVIDIA RTX3090 24 GB. The training processes are shown in Figure 6.

This study uses various online data augmentation methods in training to improve the robustness and suppress the negative impact of low-quality images. The methods and parameters used are listed in Table 2. Only one category lesion label is reserved when training an SDM. Others are set to empty as negative samples. When training an MDM, all labels are reserved.

These models are trained from weights pretrained on the COCO dataset [24]. Using pretrained weights in endoscopic image analysis can improve the accuracy and save training time [25, 26]. All layers are not frozen. The initial learning rate is 0.01. The warmup strategy [27] is adopted to decay the learning rate to 0.001 in the form of cosine. The optimizer uses SGD momentum, and the momentum parameter is set to 0.937. This study uses Box loss, Conf loss, and Class loss to optimize the model. Box loss is calculated based on CIoU [28] written as Equation (2). Conf loss and Class loss are calculated by cross-entropy written as Equation (3). Since the SDMs do not judge the lesion category, their Class losses are always set to 0. Due to the large value of Box loss in training, its weight is adjusted to 0.1. The weights of the other loss functions are 1.0 to make the training process smoother. This study uses mini-batch to set the batch size as 72 to obtain a better training effect. Under the above settings, these models are close to convergence after training for 1000 epochs.

(2) $$\begin{array}{c} \left\{\begin{array}{c} {\text{Loss}}_{\text{Box}}=1-\text{IoU}+\frac{\rho^{2}\left(b,b^{gt}\right)}{c^{2}}+\alpha v,\\ \text{IoU}=\frac{\text{Box}\cap \text{Bo}{\text{x}}^{gt}}{\text{Box}\cup \text{Bo}{\text{x}}^{gt}},\\ \alpha =\frac{v}{1-\text{IoU}+v},\\ v=\frac{4}{\pi^{2}}{\left(\arctan\frac{w^{gt}}{h^{gt}}-\arctan\frac{w}{h}\right)}^{2}, \end{array}\right. \end{array}$$

(3) $$\begin{array}{c} \left\{\begin{array}{c} {\text{Loss}}_{\text{Conf}/\text{Class}}=\text{mean}\left\{l_{1},\cdots l_{n}\right\},\\ l_{n}=-\left(y_{n}*\log\left(p_{n}\right)+\left(1-y_{n}\right)*\log\left(1-p_{n}\right)\right), \end{array}\right. \end{array}$$

where the Box^*gt*^ and Box are the bbox of ground-truth and prediction, respectively. *ρ*^2^(*b*, *b*^*gt*^) is the distance between the centre points of the Box^*gt*^ and Box. *c* is the diagonal length of the smallest box covering the Box^*gt*^ and Box. *w*^*gt*^ and *w* are the width of the Box^*gt*^ and Box. *h*^*gt*^ and *h* are the height of the Box^*gt*^ and Box, respectively. *y*_*n*_ and *p*_*n*_ are the label and prediction, respectively.

The article "Efficient Synchronous Real-Time CADe for Multicategory Lesions in Gastroscopy by Using Multiclass Detection Model" was published in 2022. Journal: Biomed Res Int.

### 2.5. Metrics

This study uses multiple objective metrics to evaluate accuracy and speed performance. The precision, recall, and mAP are used to evaluate the accuracy, and the frame per second (FPS) is used to evaluate the detection speed.

(4) $$\begin{array}{c} \text{Presicion}=\frac{\text{TP}}{\text{TP}+\text{FP}}, \end{array}$$

(5) $$\begin{array}{c} \text{Recall}=\frac{\text{TP}}{\text{TP}+\text{FN}}, \end{array}$$

(6) $$\begin{array}{c} \text{mAP}=\overset{\text{confidence}\_\text{threshold}=1}{\underset{\text{confidence}\_\text{threshold}=0}{\sum }}\text{P}\text{resicion}\times \text{Recall}, \end{array}$$

where TP, FP, and FN are true positive, false positive, and false negative, respectively. When IoU ≥ 0.9, the prediction is considered to have detected a lesion.

## 3. Results

### 3.1. Multicategory Lesion Detection Performance

The models with the highest accuracy on the validation set were selected to test on the test set to examine the performance of MDS, MPDS, and MSDS. These systems were run on an NVIDIA TITAN V 12 GB to simulate a PC workstation. The input image was scaled to 640 × 640 by padding, and the batch size was set to 1.

In the test, the detection speed of the MDS is 47 FPS, the latency is 0.04 s, the MPDS is 17FPS and 0.07 s, and the MSDS is 13FPS and 0.1 s. Therefore, only the MDS can run in real-time on a PC workstation. The load of running MDS is approximately 55% on the GPU and 100% on one CPU core, while the MPDS is 80% on the GPU and 65% on four CPU cores, and the MSDS is 65% on the GPU and 100% on one CPU core. It can be observed that the MDS and MSDS need similar hardware resources, but the MPDS needs many times. For MPDS, the hardware pressure and speed lower than the theory may be due to other hardware bottlenecks.

The article "Efficient Synchronous Real-Time CADe for Multicategory Lesions in Gastroscopy by Using Multiclass Detection Model" was published in 2022. Journal: Biomed Res Int.

The accuracy of the model used in the system represents the system's accuracy, as shown in Table 3. For all lesions, MDM has higher accuracy with 98% precision, 89% recall, and 90.2% mAP, whereas that of SDM is 95.5%, 88.5%, and 88.3%, respectively. The accuracies of the two types of models for GIST and polyp are similar. However, the accuracy of MDM is significantly better for the other two categories of lesions, especially in cancer.

For GIST, polyp, and ulcer, the MDM has achieved over 97% precision and over 94% recall, which are extremely high. The model can detect some targets missed in the annotation for these categories, as shown in Figure 7. However, MDM and SDM have a low recall for cancer with many false detections, as shown in Figure 8(a). The reason may be that cancer has more complex features than the others to be learned in a similar number of lesions in the training set. The other three categories have only a negligible number of missed predictions. Their features of which are usually quite different in the dataset, as shown in Figures 8(b)–8(d).

This study also evaluated the performance of MDM on different size targets defined in the “Dataset” section, as shown in Figure 9. It can be observed that the model has high accuracy for different size lesions. However, the model has higher accuracy for larger targets, which may be because larger lesions contain more features and are therefore easier to be detected.

### 3.2. Performance Comparison of Different YOLO Model Designs

In addition to YOLOv5x, this paper compared the performance of YOLOv5l, YOLOv4 [23], and YOLOv3-SPP based on MDS. The training and testing are the same as the “Training Strategy for the Lesion Detection Model” section, and the results are listed in Table 4. It can be found that the model based on YOLOv5x is significantly better than others in accuracy and can also be run in real-time. YOLOv5x can provide better detection capabilities.

### 3.3. The Influence of Train Image Number

The number of training images affects the accuracy and robustness of the deep learning model significantly. It may be one of the reasons why the model cannot detect cancers better. However, its impact needs to be clarified. This study explored the impact of the YOLOv5x based on MDS by setting the number of each lesion train image to *n* (*n* = 500, 1000, 1500, 2000, 2500, 3000, and 3500). Other settings are the same as above. The results are shown in Figure 10. It can be found that the number of training images affects different metrics of different lesions differently. For all lesion categories, the number of images hardly affects the precision after exceeding 2500 for each category. After exceeding 2000 images, other accuracy metrics improve negligibly for GIST, polyp, and ulcer but continue rising significantly for cancer. It supports the previous assumption that cancers have more complex features to be learned, making the number of training images insufficient.

The article "Efficient Synchronous Real-Time CADe for Multicategory Lesions in Gastroscopy by Using Multiclass Detection Model" was published in 2022. Journal: Biomed Res Int.

## 4. Discussion

For multicategory lesion detection, this study proposes and establishes a synchronous real-time CADe system using MDM basing YOLOv5 named MDS and two joint detection systems with multiple SDMs named MPDS and MSDS. MDS can detect cancers, GISTs, polyps, and ulcers from single images with 98% precision, 89% recall, and 90.2% mAP better than MPDS and MSDS. MDS significantly outperforms MPDS and MSDS by achieving 47 FPS with 0.04 s delay on a PC workstation. It is the only one in three systems realizing online detection. The results indicate that using MDM is more meaningful and efficient for costly labelled endoscopic images. This study also explores the influences of the model design and the training image number on the MDS performance.

The existing works [15, 29] about multicategory lesion detection mostly focus on intestinal lesions and lack of detailed study of performance. Compared with them, this study achieves real-time and more accurate detection on a large and complicated dataset and studies some factors that affect performance. The performance comparison of the MDM and SDMs is also a novelty.

The model structure used in all systems is identical to facilitate the performance comparison. Modifying the structure of SDMs may improve the speed or accuracy. However, it is not easy to improve both simultaneously. If SDM uses a more efficient structure, the model can be easily modified and trained on a dataset for multicategory lesion detection. In summary, compared with the systems combining multiple SDMs directly, the advantages of the CADe system with an MDM are comprehensive in both accuracy and speed.

Better speed is an expected advantage, but the higher accuracy is worth discussing. It is generally believed that a binary classification is easier than classifying more categories. However, the MDM is more accurate in the test, which may be due to some similar features of different lesion categories interfere with the SDM. This makes it difficult to judge whether these lesions belong to the target or not. The MDM eliminates the interference as much as possible through multicategory label supervision. It is similar to the auxiliary learning [30] for each category.

The dataset used is designed as a quantity balance of multiple lesion categories, which can eliminate the preference of models and fairly evaluate the detection performance of different categories. However, there should be differences in the distribution of four diseases in practice. This will not affect the conclusion of system designs from a technical perspective shown in this paper; however, it may affect the CADe performance in the clinic. As far as we know, there is a lack of research on the distribution of these lesions under gastroscopy, and the existing works, including the clinical studies of CADe, have not considered it. Therefore, it is difficult to design a dataset close to clinical distribution at present. In the future, if more extensive and large-scale clinical image data can be obtained in subsequent research, we will further explore the impact of lesion distribution on CADe performance from a clinical perspective.

The article "Efficient Synchronous Real-Time CADe for Multicategory Lesions in Gastroscopy by Using Multiclass Detection Model" was published in 2022. Journal: Biomed Res Int.

## 5. Conclusions

The constructed system can run on limited hardware and detect multicategory lesions accurately and synchronously in real-time. It can further expand the application of CADe in clinic and more efficiently use expensive-labelled medical images. We expect that this work will be a pioneering reference for future studies and researchers. The system can detect GISTs, polyps, and ulcers with extremely high accuracy, and the next step will be to examine its clinical effectiveness. The ways of improving the accuracy of cancer detection will also be explored in future works. In addition, we also hope to improve clinical applicability by detecting more categories or adding new features.

## Figures and Tables

**Figure 1:** Examples of low-quality images in the dataset. The formats of images are various, and there may be various artefacts, such as highlights and blur. The aspect ratios are also not the same.

**Figure 2:** The distribution of different target sizes in the dataset.

**Figure 3:** The number of different lesion categories in the dataset. (a) Training set. (b) Validation set. (c) Test set.

**Figure 4:** The synchronous multicategory lesion detection system for gastroscopy. The system is designed to run with limited hardware resources.

**Figure 5:** Structure of the lesion detection model based on YOLOv5. All models in this paper use the same design.

**Figure 6:** The training processes of detection models (a) MDM for MDS and (b) SDM for MPDS and MSDS.

**Figure 7:** MDM can detect some unannotated lesions. The first line is the label, and the second line is the model prediction.

**Figure 8:** Typical detection failure examples of each lesion category. The lesion in (a) is labelled as cancer which is detected as an ulcer because of the vitiligo. The lesions labelled in (b–d) are false positive.

The article "Efficient Synchronous Real-Time CADe for Multicategory Lesions in Gastroscopy by Using Multiclass Detection Model" was published in 2022. Journal: Biomed Res Int.

**Figure 9:** The accuracy of MDM for different size target lesions. The target size is bigger, and the accuracy is higher.

**Figure 10:** The effect of the number of training images on MDS accuracy metrics of each lesion category. The effects on the precision, recall, and mAP are shown in (a), (b), and (c), respectively.

**Table 1:** The number of images and lesions in the dataset.

Illusion	Cancer	GIST	Polyp	Ulcer	Negative sample
Number of images	6238	6239	6227	6207	6206
Number of lesions	7483	6239	7183	6336	—

**Table 2:** Data augmentation parameters in training.

Augmentation	Parameter
Transformation in HSV colour space	Transform range in hue: ±1.5% Transform range in saturation: ±70% Transform range in value: ±40%
Translation	Range: ±10%
Scale	Range: ±50%
Flip	Probability of flip up-down: 50% Probability of flip left-right: 50%
Mosaic [23]	Number of images: 4

**Table 3:** Detection performance of all lesion detection models.

	Precision		Recall		mAP	
Model	MDM	SDMs	MDM	SDMs	MDM	SDMs
All	**98%**	95.5%	**89%**	88.5%	**90.2%**	88.3%
Cancer	**95.4%**	91.7%	**66.3%**	63.7%	**67.3%**	62.9%
GIST	**99.9%**	98.5%	96.9%	**97.9%**	**98.7%**	98.6%
Polyp	**99.3%**	97.5%	**98%**	**98%**	**99%**	98.3%
Ulcer	**97.5%**	94.3%	**94.8%**	94.6%	**96%**	93.4%

**Table 4:** Performance of different YOLO model designs.

Model	Precision	Recall	mAP	FPS
YOLOv5x	**0.985**	0.885	**0.898**	47
YOLOv5l	0.903	**0.887**	0.881	51
YOLOv4	0.897	0.843	0.826	54
YOLOv3-SPP	0.879	0.831	0.802	69

## Data Availability

The data used to support the findings of this study are available from the corresponding author upon request.
